# Machine Learning-Based Multimodel Computing for Medical Imaging for Classification and Detection of Alzheimer Disease

**DOI:** 10.1155/2022/9211477

**Published:** 2022-08-12

**Authors:** Fatemah H. Alghamedy, Muhammad Shafiq, Lijuan Liu, Affan Yasin, Rehan Ali Khan, Hussien Sobahi Mohammed

**Affiliations:** ^1^Applied College, Imam Abdulrahman Bin Faisal University, Dammam, Saudi Arabia; ^2^School of Artificial Intelligence, Neijiang Normal University, Neijiang, Sichuan, China; ^3^School of Software, Tsinghua University, Beijing 100084, China; ^4^Department of Electrical Engineering, University of Science & Technology, Bannu (28100), Pakistan; ^5^University of Gezira, Wad Medani, Sudan

## Abstract

Alzheimer is a disease that causes the brain to deteriorate over time. It starts off mild, but over the course of time, it becomes increasingly more severe. Alzheimer's disease causes damage to brain cells as well as the death of those cells. Memory in humans is especially susceptible to this. Memory loss is the first indication of Alzheimer's disease, but as the disease progresses and more brain cells die, additional symptoms arise. Medical image processing entails developing a visual portrayal of the inside of a body using a range of imaging technologies in order to discover and cure problems. This paper presents machine learning-based multimodel computing for medical imaging for classification and detection of Alzheimer disease. Images are acquired first. MRI images contain noise and contrast problem. Images are preprocessed using CLAHE algorithm. It improves image quality. CLAHE is better to other methods in its capacity to enhance the look of mammography in minute places. A white background makes the lesions more obvious to the naked eye. In spite of the fact that this method makes it simpler to differentiate between signal and noise, the images still include a significant amount of graininess. Images are segmented using the *k*-means algorithm. This results in the segmentation of images and identification of region of interest. Useful features are extracted using PCA algorithm. Finally, images are classified using machine learning algorithms.

## 1. Introduction

A single image is capable of communicating more than just one single word. When making a decision, the information that is represented visually is always given the most importance, regardless of the other information that may be accessible. The importance of image processing and the applications it has fostered over the course of the last several decades has skyrocketed in a number of different academic subfields. The proliferation of different imaging techniques has been a driving force behind the expansion of image processing as a field. The field of digital image processing is branching out into a variety of new subfields of research, one of which being medical image processing. It is a subfield of radiology in which information collected from a patient's medical imaging is analyzed in order to establish whether or not the individual in question is suffering from a disease. Inside of a person's body is where the vast majority of diseases manifest themselves in people. Some examples of these diseases are brain tumors, Alzheimer's disease, breast cancer, lung cancer, and cardiovascular disease. The ability to easily diagnose and treat these conditions is made possible by medical image processing [1]. Multimodel computing is efficient in Alzheimer disease detection. Multimodel computing is useful in many medical applications like lung cancer detection, breast cancer detection, and medical image classification and detection.

Alzheimer's disease is now the primary research interest (AD). Alzheimer's disease is an example of a kind of brain disorder. Some of the most common types of medical imaging are positron emission tomography (PET), positron X-ray tomography (X-ray), computed tomography (CT), ultrasound, and magnetic resonance imaging (MRI). The circumstances of the patient are what guide the selection of the appropriate imaging technique. When diagnosing a patient with a bone problem, it is a common practice to take x-rays of the affected area of the patient's body. The diagnosis of Alzheimer's disease is the focus of the research being conducted right now, which makes use of the magnetic resonance image processing [2].

The medical needs of almost every person in this nation are met by the healthcare system provided by the pharmaceutical sector. The great majority of conditions that affect the human health are due to dysfunctions that occur inside the body's organs and tissues. Medical image processing entails developing a visual portrayal of the inside of a body using a range of imaging technologies in order to discover and cure problems [3]. This may be done via the use of computer software. The discipline of medical image processing, which is a subfield of image processing that contributes to the improvement of public health, has a number of challenges.

The magnetic resonance imaging (MRI) technique is a noninvasive medical imaging method that works by producing the images of inside organs, bones, and other human tissues via the use of high magnetic fields and radio waves. The proton magnetic resonance imaging (MRI) scanner makes use of a strong magnetic field in order to arrange the hydrogen atoms' protons within the body. After that, radio waves are used to spin the protons. After the radio waves have been turned off, the protons will realign themselves by producing new radio waves on their own. This piece of equipment is capable of picking up radio waves and producing an image of them. Magnetic resonance imaging, more often known as MRI, is the technique of choice for situations in which high-resolution images are needed, such as when abnormalities of the brain are being diagnosed. Using this strategy, one may be able to prevent exposure to radiation with a high energy level [4].

By altering the order in which the radio waves are received, various images may be produced. The repetition time refers to the amount of time that has passed between the two successive radio wave sequences that have been applied to the same slice (TR). It is possible to differentiate between the various tissues by using their respective relaxation times. Both T1 and T2 relate to relaxation times in the longitudinal and transverse axes, respectively, as well as relaxation durations in spin lattice and spin-spin lattices. Additionally, T1 and T2 refer to relaxation periods in spin-spin lattices. The time constant T1 determines the pace at which the stimulated protons return to their original state of equilibrium. T2 is the most important variable to consider when attempting to compute the rate at which the protons approach equilibrium or become out of phase with each other. MRI images may also be classified according to their sequences using terms such as T1-weighted and T2-weighted MRI. It is possible to differentiate between T1- and T2-weighted photographs by using the cerebrospinal fluid (CSF) that is found in the brain. The cerebrospinal fluid (CSF) appears black in T1-weighted imaging, but it appears bright in T2-weighted pictures.  Figure 1 displays an image that is weighted T1 as well as a photo that is weighted T2 [5].

Dr. Alois Alzheimer was the one who first recognized the symptoms of Alzheimer's disease (AD) in 1906. Each year, more than two million people in World are given a diagnosis of Alzheimer's disease [6]. It is a disease that causes the brain to deteriorate over time. It starts off mild, but over the course of time, it becomes increasingly more severe. Alzheimer's disease causes damage to brain cells as well as the death of those cells. Memory in humans is especially susceptible to this. Memory loss is the first indication of Alzheimer's disease, but as the disease progresses and more brain cells die, additional symptoms arise. These include shifts in mood and behavior, difficulties communicating, and problems remembering the names of known people, places, or recent events. People who have Alzheimer's disease may eventually reach a point when they are unable to do the tasks required of them on their own. They put their whole well-being in the hands of another person. This is due to the fact that brain changes that accompany normal ageing may bring about memory loss. To put a stop to the progression of Alzheimer's disease (AD), however, it is essential to diagnose the condition at an early stage. Even though there is currently no cure for Alzheimer's disease, early discovery of the condition might potentially reduce or stop the progression of the illness.

Alzheimer's disease (AD) is characterized largely by the death of nerve cells and tissues in the brain, which ultimately leads to a reduction in brain volume. The brain is both an essential component of the nervous system as well as one of its most intricate components. The human brain is made up of three different parts: the cerebrum, the brainstem, and the cerebellum. The largest and most complex part of the neurological system, the cerebrum is located at the front of the skull. This part of the brain is involved in a broad range of mental functions, such as memory, reasoning, problem solving, emotional regulation, and the perception of sound and light. There are two hemispheres of brain in the cerebrum: left and right. The grey matter of the cerebral cortex, the outermost layer of the cerebrum, dominates this region. In the brain's cortex, which is made up of several layers, there are billions of nerve cells. “White matter” is a lengthy nerve fibre that connects the different parts of the brain together and is often referred to as such. One of the early warning signs of Alzheimer's disease is a reduction in grey matter in the cerebral cortex. The hippocampus and basal ganglia are only two examples of the many subcortical structures found inside the cerebrum. The four lobes of the cerebrum are the frontal lobe, temporal lobe, occipital lobe, and parietal lobe. As Alzheimer's disease progresses, the temporal lobe of the brain is most often afflicted. Other brain areas will also begin to degenerate as the illness progresses. Both movement coordination and the maintenance of balance are crucial functions of the cerebellum, which resides immediately below the cerebrum. Several of the body's autonomic processes, including digestion, respiration, heart rate, and temperature, are controlled by the brainstem, which lies underneath the cerebral cortex and directly in front of the cerebellum. The cerebrum, which is positioned at the top of the skull, is the primary target of Alzheimer's disease (AD) [7].

The magnetic resonance imaging (MRI) technique is helpful for providing a dynamic diagnostic of the structure and volume of the brain. In order to make an accurate diagnosis, it is essential to have the capability of recognizing quick changes in the brain utilizing dynamic analysis. Magnetic resonance imaging, sometimes known as an MRI, is a technique that is frequently used for the purpose of precisely diagnosing Alzheimer's disease in its initial stages. Changes in the hippocampus and entorhinal cortex will be seen in the reports generated by MRIs performed on people with Alzheimer's disease. Because of the possibility of mistakes and inaccuracies introduced by the involvement of humans in the process, it is necessary to use more efficient alternatives such as automated systems. MRI features and machine learning algorithms are used to make an automatic diagnosis of Alzheimer's disease.

Literature review section contains a review of modern techniques for Alzheimer disease detection. Methodology section presents machine learning-based multimodel computing for medical imaging for classification and detection of Alzheimer disease. Images are acquired first. MRI images contain noise and contrast problem. Images are preprocessed using CLAHE algorithm. It improves image quality. Images are segmented using the *k*-means algorithm. This results in the segmentation of images and identification of region of interest. Useful features are extracted using PCA algorithm. Finally, images are classified using machine learning algorithms. Result section contains details related to input data set and results obtained by various machine learning algorithms. Conclusion section contains major contributions of the research article.

### 1.1. Medical Image Processing

The phases of medical image processing are image preprocessing, image segmentation, and feature extraction and classification.

### 1.2. Preprocessing

Preprocessing, often known as augmentation, is the first step in the medical image processing workflow [8]. Image enhancement, often known as preprocessing, is the process of improving an image's quality before it is utilized in following processing steps. This allows the image to be put to better use. This method is used to improve the picture quality since it is possible that an inaccurate diagnosis might result from an inaccurate image. Before they can be used in the diagnostic process, medical images often need some kind of update. The removal of noise, improvement of contrast, and “skull stripping” are three of the most common MRI image modifications.

There will always be some level of noise in an image, regardless of the method used to shoot the picture or the gear that was used. The process of reducing unwanted noise from an image is referred to as noise reduction. Noise may be reduced using a number of filtering techniques, many of which are available via digital image processing.

The process of boosting the dynamic range of an image's intensity values is referred to as “contrast enhancement,” and it is one of many methods that can be used to improve the contrast of an image. The image's primary components become more distinguishable from the background when the contrast has been increased.

In a brain MRI, it is possible to view tissues that are not part of the brain, such as the skull, skin, fat, muscle, and the neck. The existence of these non-brain tissues makes it difficult to do further study on those tissues. Skull stripping [3] is the process that is utilized to remove non-brain material prior to continuing the examination of the patient. In this study, skull stripping was accomplished by the use of entropy-based thresholding in conjunction with several morphological methods.

### 1.3. Segmentation

In the field of medical image processing, segmentation [9] is a technique that is used to separate the diseased region from the rest of the image. It does this by using aspects like as intensity or texture to separate an image into discrete pieces depending on how similar they are to one another. It is possible to make use of the divided region of interest in order to readily extract crucial information for the purpose of sickness detection.

Using approaches that are based on a threshold, images may be segmented. It is a translation from binary to pictures. In this method, every pixel in the image is either completely black or completely white. In a digital picture, the intensity of a pixel is compared to a threshold, which is a constant value denoted by the letter “T.” Based on this value, the pixel is either replaced with a white or a black pixel.

If you use the strategy of region-based segmentation, you may be able to find regions that have certain qualities in common with one another. It does this by slicing the image up into distinct subregions, none of which can share the same characteristics with one another. It is possible to divide it into two groups, namely, the expansion of regions and the division and combination of regions. In the method for growing regions, a seed point is utilized, and the area grows outward from that point by connecting pixels that are near to the seed and have properties with the seed itself. The starting point might be one or many seed points, depending on the situation. Using the Split and Merge method, first some random bits are divided into, and then they may be combined and/or split in an attempt to generate unique regions in the image that are of a similar nature to one another.

Edge-based segmentation software often uses this method, which involves dividing an image into sections depending on the edges or boundaries that it has. The field of image processing provides a wide number of options for finding edges. Methods for locating edges often focus on identifying discontinuities or changes in intensity. The intensity levels of an image item rapidly change as they get closer to the picture's borders.

K-means clustering is the method that is used the majority of the time in the process of medical image segmentation. During the clustering technique, the image is cut up into distinct groups or clusters that do not overlap with one another. In this image, there are a few different clusters, and each of these clusters has its own unique set of reference points to which each pixel is assigned. The k-means clustering method utilizes *k* reference points and results in *k* distinct groups.

### 1.4. Feature Extraction

In order to facilitate the process of sickness diagnosis, a technique known as feature extraction is used to glean important and pertinent information from a sectioned off region of interest. The recovered characteristics have a direct bearing on the level of accuracy that may be achieved while diagnosing a disease. If the traits that are produced from the classification are employed appropriately, it is possible that more informed judgments may result. When it comes to the processing of medical images, shape and size are the most crucial components. Because Alzheimer's disease changes the size and shape of the brain, the classification results of brain MRIs performed to diagnose Alzheimer's disease may be affected as a result.

### 1.5. Classification

Image processing often continues with categorization as the next step after the extraction of features. Both the classifier that was applied to the image in order to classify it and the recovered features from the image itself are directly responsible for the result of the classification. When the class of an image cannot be determined, the classifier will give the picture a label. In this instance, the classification for the class might be either normal or abnormal (with disease). In the field of medical image processing, two of the classifiers that are used most often are the k-nearest neighbor and the support vector machine [10].

For the purpose of data classification, a strategy known as the k-nearest neighbor algorithm (k-NN) is used. In the k-NN classification system, the majority of an image's neighbors decide whether or not an image should be considered normal or abnormal. The image gets filed away in a particular classification according to which of its *k* immediate neighbors it has the most characteristics with. A positive integer that goes by the name *k* is one of the numbers that comes up most often.

A binary classifier is a technique that is recognized by the acronym SVM (which stands for support vector machine). It is possible to predict the class of each feature vector by utilizing a feature vector as the input. The approach in question creates two categories, which are referred to as normal and abnormal, and places a significant gap between them. Based on the data that is at hand, it is clear that the SVM classifier generates very good results when it is coupled with an appropriate kernel. The equation for the hyperplane of the linear SVM is as follows:

(1) $$\begin{array}{c} ww.ll+bb=00, \end{array}$$

where, *b* = real number, *w* = normal vector to the hyperplane, *l* = feature vector.

Artificial neural networks, also known as ANNs, are often used in the process of classifying medical pictures for the purpose of disease diagnosis. The functioning of the ANN is quite similar to that of the human brain. By looking at a collection of pictures that have already been labelled, it is able to acquire the knowledge necessary to make an accurate estimate about the category that an image belongs to. Artificial neurons, which are the building blocks of an ANN, are designed to mimic their natural counterparts in the human brain. Neurons are connected to one another along their edges. Weights may be assigned to neurons and edges, and these can be altered at any point throughout the learning process. The majority of artificial neural networks are constructed with three layers: an input layer, a hidden layer, and a final layer that is responsible for outputting the signal. It is possible that there is only one hidden layer, that there are numerous hidden levels, or that there are none at all. Weights are adjusted inside a layer that is concealed from view until the desired result is obtained.

### 1.6. Literature Survey

#### 1.6.1. Literature Review of Image Preprocessing Algorithms

Priyanka and Balwinder [11] proposed the possibility of using a method known as the Median Filter in order to get rid of salt and pepper noise as well as Poisson noise in photographs. For instance, the output intensity value of the pixel that is to be processed is made by sliding a window across the image. This value is then determined by using the median intensity of the pixels that are included inside the window to calculate the value. In addition, the median filter maintains the borders of a picture while simultaneously minimizing the amount of random noise. The values of every pixel are permanently set to the median of the values of the pixels that are immediately around them. After that, it is put to use to get rid of these noises, and after that, the bounding box approach is carried out to find the tumor.

Yousuf and Nobi [12] state that the research into the creation of order statistics filters has resulted in the invention of a simple solution that is both efficient and effective for cutting down on the amount of noise present in medical images. As can be seen in the above illustration, the median and mean filters are used in order to get the pixel value of a picture that is free of noise. In addition, it may be used to lessen the appearance of visual artefacts such as Rician noise.

Jaya et al. [13] came up with the idea for the weighted median filter. The use of a weighted median filter for denoising allows for the reduction of high frequency components as well as the removal of salt and pepper noise from images without causing the edges to become distorted. Additionally, it may be used to extract each pixel from a window of pixels that is 3 by 3, and then analyze the mean value of the foreground and background pixels, as well as the contrast value. The background noise in a picture may be removed using an anisotropic filter that was created by Ramalakshmi and Chandran [14].

Comparisons were then made between the wavelet denoising and the Gaussian smoothing techniques [15]. In the steps leading up to the reconstruction of MR images, a wavelet-domain Wiener-filtering technique was used [16]. However, because of the underlying wavelet structure, the wavelet-based techniques that are often utilized have the potential to result in considerable artefacts being introduced into the processed images. One of the most prevalent approaches to denoising that is now accessible is called a maximum posteriori estimate methodology. Rician noise is taken into consideration in these approaches by the use of both a data probability term and a spatial smoothing prior [17]. Empirical Bayes was used by Awate and Whitaker [18] for the MRI denoising process. The Markov Probability Density Function (PDF), which is used as a prior in Bayesian estimation, is used to do an analysis of the distortions that are present in the data.

#### 1.6.2. Literature Review of Feature Extraction Algorithms

Either image segmentation or the registration of a brain Atlas over the image may be used to count the voxel values in important anatomical locations. This can be done either manually or automatically. In spite of these challenges, the structural parcellation of the brain may not be able to adjust to the effects of the illness.

To begin, Khajehnejad et al. [19] employed voxel morphometry analysis to extract from actual MRI volumes and Gray Matter (GM) segmentation volumes some of the most likely AD-relevant elements of brain imagery. These volumes were segmented based on grey matter. The characteristics that set a healthy brain from one afflicted by Alzheimer's disease must be included into the characteristics of the features. After that, a dimension reduction using Principal Component Analysis (PCA) is carried out on the collected features in order to conduct an analysis that is not only quicker but also more accurate. In order to make use of the returned features, a hybrid manifold learning framework has been proposed here. This framework brings feature vectors into a subspace.

Assessment of the cortical thickness that is quick, accurate, and completely automated has been created by Querbes et al. [20]. There may be a connection between the existence of histopathological validated anomalies and the progression of cortical atrophy, which is evaluated by the cortical thickness. It is possible to make adjustments to the volume in this way by utilizing the estimated total brain volume by Cuingnet et al. [21]. Cortical thickness testing provides the chance for results that are less dependent on the operator, in contrast to hippocampal volume measurement, which is highly dependent on the individual doing the test by Higdon et al. [22]. Those with higher levels of education and more severe brain damage have a greater propensity to conceal indications of dementia due to their cognitive reserve. This may be perplexing to people who are not acquainted with the condition since it occurs less often in people with a higher levels of education.

Using ROI-based techniques, one or more essential components of the brain, such as the cingulum, the corpus callosum, and similar structures, may be characterized. Studies have indicated that the development of neurodegeneration in Alzheimer's disease (AD) affects the regions of the brain that are situated in the limbic and neocortical areas, as well as the temporal and temporal lobes of the brain. Additionally, the temporal and temporal lobes of the brain are affected. The atrophy of the medial temporal region, and in particular the atrophy of the hippocampi, is generally recognized as a sensitive biomarker of Alzheimer's disease (AD) [23]. As a consequence of this, hippocampi have been employed in a number of studies as a biomarker for early-onset Alzheimer's disease.

In addition, Sakthivel et al. [24] incorporated not just the information that can be found in text and photographs, but also the direct input from the doctor. It is possible for a feature to have coefficients that match up to an image spectral transform, such as Fourier or Discrete Cosine Transform (DCT) coefficients, statistics on picture gradients, and other such things. Two characteristics that are utilized to characterize the brain images are called Local Binary Patterns (LBPs) and Discrete Cosine Transforms (DCT).

Researchers have successfully extracted three separate features from the MR scans of the brain for the very first time by combining the grey matter volume, the Gray-Level Co-Occurrence Matrix (GLCM), and the Gabor feature. This achievement marks a first. The results of the experiments indicate that a greater performance may be accomplished by the multifeature fusion of these characteristics, which may gather both 2D and 3D information on brains. This can be accomplished by combining the features of many brain scans. The researchers Agarwal and Mostafa [25] employed visual image similarity as a tool to assist in the early identification of Alzheimer's disease. It displays how well the brain images may be categorized depending on the information provided by the user. Calculations of Circular Harmonic Functions and Scale Invariant Features Transform (SIFT) descriptors are performed close to the hippocampus, same as in a prior work [26]. After that, a number of classification schemes are used in order to make comparisons between the photographs.

#### 1.6.3. Literature Review of Classification Methods

Because there are so many voxels in the brain, the qualities that may be deduced from the combination of voxels are quite specific and precise. LDA is a well-known method for reducing the dimensions of a problem; another name for this method is the Fisher linear discriminant (FLD). As an example, linear discriminant analysis (LDA) makes use of a linear discriminant function to locate low-dimensional linear combinations of variables that provide the most accurate description of the data. In order to do this, the between-class scatter matrix is made larger while the within-class scatter matrix is made smaller [27].

A technique based on machine learning that was developed by Long et al. can differentiate between patients suffering from moderate cognitive impairment (MCI) and healthy older persons. It is also possible to use this method to forecast whether or not a patient diagnosed with MCI would eventually develop Alzheimer's disease (AD). After this phase, a symmetric diffeomorphic registration, an embedding approach, and a learning method for determining the distance between the subjects are available. These results were obtained when the amygdala and/or hippocampus were used as the area of interest (ROI): 96.5 percent for mild AD identification, 91.74 percent for progressive MCI differentiation, and 88.99 percent for classification of the two types of MCI. By using the macroscopically distinct shapes that occur in each pair, this technique has maximized its differentiation potential.

Zhao et al. [28] invented the Iterative Trace Ratio (iITR) to address the TR-LDA (Trace Ratio Linear Discriminant Analysis) issue for dementia diagnosis. iITR outperformed PCA, LPP, and the Maximum Margin Criterion in terms of outcomes. [Reference required] (MMC). Image features used to distinguish between AD and FTD in LDA were compressed using the Partial Least Squares (PLS) approach by Horn et al. [29]. The accuracy, sensitivity, and specificity of the SPECT pictures obtained by the researchers were all over 84%.

Those classifiers that come from the Nave Bayes theorem are in the same family as other probabilistic classifiers since they make the assumption of feature independence. Decision models for Alzheimer's disease (AD), moderate cognitive impairment (MCI), and neurological dementia (NC) were developed by Seixas et al. [30]. In the end, they concluded that the Bayesian network decision model outperformed several well-known classifiers, including the naive Bayes, the logistic regression model, the multilayer perceptron ANN, and the decision table. Liu and Shen [31] multifold Bayesian Kernelization approach is better at distinguishing between Alzheimer's disease (AD) and non-converter (NC) MCI, but it is less accurate at identifying MCI-converter (MCIc) and non-converter (MCIn).

SVMs allow for the construction of hyperplanes with high or indeterminate dimensions, which may then be utilized for a variety of applications, including classification and regression. Because SVMs have a lower generalization error compared to other classifiers, they are frequently used to solve pattern-classification problems with limited sample sizes [32]. There are a total of 120 subjects, with 40 ADs, 40 MCIs, and 40 NCs allocated to each of the three categories, respectively. In the beginning, each subject was subjected to filtering and normalization, and after that, K-Nearest Neighbor (KNN) or Support Vector Machine was used in order to extract a total of twelve features (SVM). It was determined that several permutations and combinations of each feature should be tried in order to uncover the best characteristics for categorizing the data. This was done with the intention of finding out which ones were the most accurate. For a random selection of test data using SVM and KNN, the results showed an accuracy of 95.833 percent on average, with SVM polynomial order three yielding the highest accuracy at 97.92 percent, and KNN with *K* = 6 and *K* = 7 yielding the lowest accuracy at 95.83 percent. It was shown that there was a high level of accuracy in classification across all three clinical groupings. The Master Characteristics of the images were extracted with the use of a quick discrete wavelet transform (DWT), and then the Principal Component Analysis (PCA) was utilized to conduct additional research on the distinguishing characteristics that were discovered (PCA). There are a total of five distinct decision models that are each given a unique subset of the key feature vectors. Models such as the J48 decision tree and KNN, Random Forest (RF), and LS-SVM with polynomials and radial basis kernels are used as part of the classification models.

The covariance method was used to study several feature correlation technologies and enhance the SVM-RFE algorithm by means of the covariance technique. This was accomplished via the usage of the covariance approach. The recently devised strategy seems to be beneficial, based on the results of analyses conducted on the publicly available ADNI database. It also suggests that using a combination of numerous features is preferable than making use of a single trait on its own.

It is possible to estimate for approximation functions that are dependent on a large number of unknown inputs by using models that are based on artificial neural networks (ANNs), which are a subset of models that are impacted by biological neural networks. They have taken the place of rule-based programming as the go-to solution for a broad variety of complicated issues, and with good reason. Standard discriminant function analysis was shown to have lower sensitivity and accuracy compared to employing an artificial neural network (ANN) for MRI-based dementia classification.

Luo et al. [33] presented a deep learning system that was built on 3D brain MRI as a way for automatically identifying the Alzheimer's disease. This system was stated as being able to do so. Convolutional Neural Network (CNN) is used in order to diagnose Alzheimer's disease (AD). One of the most important distinctions is that in the identification of AD, the three-dimensional structure of the brain is regarded to be complete, making it possible to make an accurate diagnosis. The Convolutional Neural Network (CNN) that was used in this investigation contains three consecutive sets of processing layers, two levels that are totally connected, and a classification layer. Each of the three different groups has a structure that consists of a convolutional layer, a pooling layer, and a normalizing layer. All three layers are included.

## 2. Methodology

This section presents machine learning-based multimodel computing for medical imaging for classification and detection of Alzheimer disease. Images are acquired first. MRI images contain noise and contrast problem. Images are preprocessed using CLAHE algorithm. It improves image quality. Images are segmented using the *k*-means algorithm. This results in segmentation of images and identification of region of interest. Useful features are extracted using PCA algorithm. Finally, images are classified using machine learning algorithms. Block diagram of the model is shown in Figure 2.

In order for an image to be accurately recognized, the process of background extraction has to be able to adapt to the one-of-a-kind characteristics of the particular photograph being used. Within CLAHE, the histogram is only constructed for the pixels that are immediately next to it. By imposing a “clip level” on the height of the local histogram and, therefore, the maximum contrast enhancement factor, CLAHE limits the amount of contrast alteration that may be performed. Because of this, there is noticeably less noise in the final image. CLAHE is better to other methods in its capacity to enhance the look of mammography in minute places. A white background makes the lesions more obvious to the naked eye. In spite of the fact that this method makes it simpler to differentiate between signal and noise, the images still include a significant amount of graininess [34].

Segmentation is a method that is employed in the area of medical image processing. Its purpose is to separate the diseased portion of an image from the healthy parts of the picture. It accomplishes this goal by segmenting a picture into distinct parts based on how closely those pieces resemble one another. This is done using image characteristics such as intensity and texture. It is feasible to make use of the segmented area of interest in order to quickly extract important information for the aim of diagnosing a disease. In the process of medical picture segmentation, the technique known as k-means clustering is the one that is used the vast majority of the time. During the clustering process, the picture is divided into a number of unique groups, also known as clusters, which do not overlap with one another. This picture has a few distinct clusters, and each of these clusters has its own one-of-a-kind set of reference points to which each pixel is allotted. The k-means clustering technique divides the data into *k* different groups using the *k* reference points that are provided in the process [35].

The approach known as Principal component analysis (PCA) is used in the process of feature extraction [36]. The method of principal component analysis (PCA) to reducing linear dimensions might be helpful in data analysis and compression [37]. Using this method, which involves finding orthogonal linear combinations of the attributes of the initial data set, it is possible to combine qualities that are not connected with one another.

A binary classifier is a technique that is recognized by the acronym SVM (which stands for support vector machine). It is possible to predict the class of each feature vector by utilizing a feature vector as the input. The approach in question creates two categories, which are referred to as normal and abnormal, and places a significant gap between them. Based on the data that is at hand, it is clear that the SVM classifier generates very good results when it is coupled with an appropriate kernel [37]. SVM works better with RBF function. The equation for the hyperplane of the linear SVM is as follows:

(2) $$\begin{array}{c} ww.ll+bb=00, \end{array}$$

where, *b* = real number, *w* = normal vector to the hyperplane, *l* = feature vector.

The process of categorizing medical images for the goal of illness detection often makes use of artificial neural networks, which are sometimes referred to by their acronym, ANNs. The way in which the ANN works is quite comparable to the way in which the human brain does. It is possible to learn the information essential to make an accurate guess about the category that an image belongs to by looking at a collection of photographs that have previously been labelled. This collection of pictures has already been classified. Artificial neurons, which are the fundamental components of an ANN, are intended to function in a manner similar to that of their natural counterparts in the human brain. Along the margins of their bodies, neurons are linked to one another. It is possible to provide weights to neurons and edges, and these weights may be changed at any time in the course of the learning process. The majority of artificial neural networks are built with three layers: an input layer, a hidden layer, and a final layer that is in charge of outputting the signal. The majority of artificial neural networks are built with three layers: an input layer, a hidden layer, and a final layer. It is conceivable that there is only one hidden layer, that there are several hidden layers, or that there are none at all. All of these outcomes are feasible. Adjustments are made to the weights that are contained inside a layer that is hidden from view until the outcome that is sought is achieved [38].

J. Ross Quinlan is the one who came up with the ID-3 technique, which is also referred to as the Iterative otomiser-3. This was the first strategy to use a dynamic decision tree as its foundation. This technique utilises a measure of information gain in addition to entropy as its primary metric. Beginning with a nodule is the first step in an iterative process that establishes an entropy value for each of the functional qualities. Under the strictest sense, data sets that have the lowest error rates are referred to be “split attributes” in the theories of entropy and “information gain” (entropy). Since there is no definitive categorization of the target classes, the algorithm must repeat through its own stages for each individual subset of data. The nonterminal nodes that make up a branch's terminal nodes are what are referred to as that branch's terminal nodes. The split attribute may be utilized to determine whether nodes inside a tree structure are not terminal since these nodes do exist [39].

## 3. Result, Analysis, and Discussion

This experiment makes use of the data gathering that was performed by OASIS [40]. In all, this dataset has 416 different samples. Machine learning strategies such as SVM-RBF, ANN, and ID3 are used while classifying the data. All forms of Alzheimer's disease, including mild Alzheimer's disease, huntington disease, and even normal MRI scans, are grouped together under the umbrella term Alzheimer's disease. The fifty pictures that make up each category were selected at random from a pool of two hundred images.

Five parameters such as accuracy, sensitivity, specificity, precision, and recall are used in this study to compare the performance of different algorithms.

(3) $$\begin{array}{c} \text{Accuracy}=\frac{\left(\mathrm{TP+TN}\right)}{\left(\mathrm{TP+TN+FP+FN}\right)},\\ \text{Sensitivity}=\frac{\mathrm{TP}}{\left(\mathrm{TP+FN}\right)},\\ \text{Specificity}=\frac{\mathrm{TN}}{\left(\mathrm{TN+FP}\right)},\\ \text{Precision}=\frac{\mathrm{TP}}{\left(\mathrm{TP+FP}\right)},\\ \text{Recall}=\frac{\mathrm{TP}}{\left(\mathrm{TP+FN}\right)}, \end{array}$$

where, TP = True Positive. TN = True Negative. FP = False Positive. FN = False Negative.

As can be shown in Figures 3–7, the SVM-RBF classifier offers the highest level of accuracy out of all of the available options for diagnosing Alzheimer's disease. ANN and Random ID3 come up at second and third place, respectively, when it comes to sensitivity, specificity, accuracy, and recall. The ANN algorithm's sensitivity and recall are much higher than those of the other classifiers. SVM-RBF is superior to the other classifiers in terms of its level of specificity.

## 4. Conclusion

Alzheimer's disease is a progressive deterioration of brain function that happens over time. It begins off not being very serious, but as time passes, it quickly escalates into a much more serious condition. Alzheimer's disease is a degenerative neurological condition that leads to both the damage and death of brain cells. Memory in humans is particularly prone to being affected by this. The initial sign of Alzheimer's disease is memory loss, but as the illness advances and more brain cells die, more symptoms emerge. Alzheimer's disease is characterized by a progressive loss of brain cells. In the field of medicine, “medical image processing” refers to the process of creating a visual representation of the internal workings of a body by using a variety of imaging technologies in order to diagnose and treat illnesses. In this study, we describe a machine learning-based multimodel computing approach for medical imaging, with the goals of classifying patients and locating Alzheimer's disease. The process begins by acquiring images. MRI imaging has noise and contrast issue. The CLAHE algorithm is used as a preprocessor for the images. It results in a higher overall picture quality. The k-means technique is used in order to separate the images. This leads to the segmentation of the pictures as well as the detection of the area of interest. Utilizing the PCA technique, useful characteristics are retrieved. In the last step, photos are categorized with the help of machine learning algorithms. SVM-RBF classifier offers the highest level of accuracy out of all of the available options for diagnosing Alzheimer's disease. ANN and Random ID3 come up at second and third place, respectively, when it comes to sensitivity, specificity, accuracy, and recall. The ANN algorithm's sensitivity and recall are much higher than those of the other classifiers. SVM-RBF is superior to the other classifiers in terms of its level of specificity.

## Figures and Tables

**Figure 1:** (a) T1-weighted MRI, (b) T2-weighted MRI.

**Figure 2:** Machine learning-based multimodel computing for medical imaging for classification and detection of Alzheimer disease.

**Figure 3:** Accuracy comparison of machine learning algorithms.

**Figure 4:** Sensitivity comparison of machine learning algorithms.

**Figure 5:** Specificity comparison of machine learning algorithms.

**Figure 6:** Precision comparison of machine learning classifiers.

**Figure 7:** Recall comparison of machine learning classifiers.

## Data Availability

The data used to support the findings of the study can be obtained from the corresponding author upon request.
